# Construction and Validation of a Lung Cancer Diagnostic Model Based on 6-Gene Methylation Frequency in Blood, Clinical Features, and Serum Tumor Markers

**DOI:** 10.1155/2021/9987067

**Published:** 2021-06-26

**Authors:** Chunyan Kang, Dandan Wang, Xiuzhi Zhang, Lingxiao Wang, Fengxiang Wang, Jie Chen

**Affiliations:** ^1^Department of Pathology, Henan Medical College, Zhengzhou, Henan Province, China 451191; ^2^Department of Breast Surgery, The Second Affiliated Hospital of Zhengzhou, Zhengzhou, Henan Province, China 450014; ^3^Department of Information and Telemedicine, The Fifth Affiliated Hospital of Zhengzhou University, Zhengzhou, Henan Province, China 450052

## Abstract

Lung cancer has a high mortality rate. Promoting early diagnosis and screening of lung cancer is the most effective way to enhance the survival rate of lung cancer patients. Through computer technology, a comprehensive evaluation of genetic testing results and basic clinical information of lung cancer patients could effectively diagnose early lung cancer and indicate cancer risks. This study retrospectively collected 70 pairs of lung cancer tissue samples and normal human tissue samples. The methylation frequencies of 6 genes (FHIT, p16, MGMT, RASSF1A, APC, DAPK) in lung cancer patients, the basic clinical information, and tumor marker levels of these patients were analyzed. Then, the python package “sklearn” was employed to build a support vector machine (SVM) classifier which performed 10-fold cross-validation to construct diagnostic models that could identify lung cancer risk of suspected cases. Receiver operation characteristic (ROC) curves were drawn, and the performance of the combined diagnostic model based on several factors (clinical information, tumor marker level, and methylation frequency of 6 genes in blood) was shown to be better than that of models with only one pathological feature. The AUC value of the combined model was 0.963, and the sensitivity, specificity, and accuracy were 0.900, 0.971, and 0.936, respectively. The above results revealed that the diagnostic model based on these features was highly reliable, which could screen and diagnose suspected early lung cancer patients, contributing to increasing diagnosis rate and survival rate of lung cancer patients.

## 1. Introduction

Lung cancer is still the leading cause of cancer death globally [1]. It is histologically composed of 85% nonsmall cell lung cancer (NSCLC) and 15% small cell lung cancer (SCLC). NSCLC can be further subdivided into adenocarcinoma, squamous cell carcinoma, large cell carcinoma, and bronchoalveolar carcinoma (BAC) [2]. The early stage of lung cancer is insidious, leading to the delayed diagnosis in the advanced stage and extremely poor prognosis of patients [3]. Due to the high incidence, high mortality, and limited treatments of lung cancer, promoting early diagnosis of lung cancer is one of the most effective ways to lower mortality and improve the prognosis of patients with lung cancer.

Early screening can effectively diminish lung cancer mortality. Existing imaging techniques such as low-dose computerized tomography (CT) screening can lessen lung cancer mortality by 20%. However, low-dose CT application for lung cancer screening is limited by the high false positive rate and high cost, and its repeated scanning will cause certain harm to the human body [4]. Although several peripheral blood protein tumor markers are capable of enhancing early diagnosis rate, such as carcinoembryonic antigen (CEA), squamous cell carcinoma antigen (SCCA), cytokeratin 19 fragment antigen (CYFRA21-1), and mucin 16 (CA125), it is unable to be promoted well in clinical practice owing to low sensitivity and specificity [5]. Hence, in the current precise treatment of tumors, it is urgent to develop novel diagnostic methods for further improving the sensitivity and specificity of early diagnosis of lung cancer. Numerous studies showed that in lung cancer, the hypermethylation modification of the CpG island in promoter regions of tumor suppressor genes, such as FHIT, p16, MGMT, RASSF1A, APC, and DAPK, leads to the occurrence of lung cancer and poor prognosis in lung cancer patients [6–8]. Methylated FHIT, MGMT, p16, and RASSF1A are underlying superior biomarkers, which can be used for lung cancer screening and auxiliary detection [9]. Abnormal methylation frequencies in the promoter regions of APC and DAPK genes lend a hand for the diagnosis of lung cancer [10, 11]. Targeted methylation sequencing of plasma cell-free DNA (cfDNA) is useful in the early diagnosis of lung cancer [12]. At present, the application of computer-assisted diagnosis of cancer is widely used, of which support vector machine (SVM) is one of the most practical classification methods. For example, the best accuracy of 94.643% and sensitivity of 94.595% obtained by the SVM classifier in testing 57 new PAT data from 19 ovarian cancer patients suggested that the SVM classifier potentiates to advance cancer diagnosis [13]. Notwithstanding the attempt to construct methylation-related models for diagnosis, few studies reported the construction of a diagnostic model based on tumor marker levels, gene methylation frequency, and clinical features by using the SVM classifier.

Based on previous studies and our investigation, we believed that the methylation of 6 tumor suppressor genes (FHIT, p16, MGMT, RASSF1A, APC, and DAPK) was associated with the prognosis of lung cancer patients. Thus, this study attempted to establish a diagnostic model for suspected lung cancer patients based on clinical features, 6-gene methylation frequency in blood, and tumor marker levels by using the SVM classifier. This model can assist in the early screening and diagnosis of patients with lung cancer, so as to unfold the lung cancer risk of suspected patients as early as possible, thereby treating patients in time and elevating their survival rate.

## 2. Materials and Methods

### 2.1. Clinical Samples

This study retrospectively reviewed 70 cases of outpatients (45 males and 25 females, 30 to 85 years old) affected by lung cancer in The Second Affiliated Hospital of Zhengzhou University and Henan Provincial Chest Hospital from 2015.03.31 to 2019.11.31. Patients in Stage I to IV who met the following criteria were included: (1) patients were diagnosed in clinical and histopathological as primary lung cancer without other organ diseases; (2) patients did not receive any previous radiotherapy, chemotherapy, or surgery before sampling. Normal clinical samples were collected from 70 healthy donors (36 males and 34 females, 32 to 81 years old) who underwent physical examination in The Second Affiliated Hospital of Zhengzhou University and Henan Provincial Chest Hospital were recruited as a control group. All of the healthy subjects had no other organ diseases. Patient's clinical profiles including age, gender, smoking history, pathological type, primary lesion, and Stage were collected. Clinical information on healthy subjects included age, gender, and smoking history. The research protocol was approved by the Medical Ethics Committee of The Second Affiliated Hospital of Zhengzhou University and Henan Provincial Chest Hospital, and all participants signed informed consent.

### 2.2. cfDNA Isolation and Purification

QIAGEN PAXgene® Blood ccfDNA Tube (Shanghai Yihui Biological Technology Co., Ltd.) was used to collect fasting venous blood (>6 mL/patient). Blood samples were centrifuged at 2000 r·min^−1^ for 15 min at 4°C. The serum was routinely isolated for tumor marker detection and cfDNA extraction, separately.

cfDNA was extracted from blood samples with GeneJET Whole Blood Genomic DNA Purification Mini Kit (Thermo Fisher Scientific) and subject to purity analysis with NanoDrop ND-1000 Spectrophotometer (NanoDrop, USA).

### 2.3. Detection of Tumor Markers

The lung cancer tumor marker levels in the serum samples were assessed with the following kits per the manufacturer's instructions. CEA kit (ab99992) and CA125 kit (ab274402) were purchased from Abcam, Cambridge, UK. CYFRA21-1 kit (Cat No.211-10) and SCCA kit (Cat No.800-10) were accessed from Sweden CanAg (Beijing). In brief, the corresponding dose of the calibrator and unknown samples were added to each microtiter plate well; then, 50 *μ*l of CONJ HRP was dispensed onto the sample, pipetting, and mixing. The plate was sealed and incubated at 37°C for 60 min, then rinsed with buffer, followed by addition of 100 *μ*l SUBS TMB and incubation at 18°C-25°C for 10-20 min. Finally, the reaction was stopped by adding 100 *μ*l of STOP, pipetting and mixing. The absorbance of each microtiter plate well at 450 nm was read with a microplate reader within 30 min. A standard curve was plotted with the standard samples in the kit. The concentration of CEA, CA12, CYFRA21-1, and SCCA in each sample was determined according to the standard curve. If the concentration of proteins was >50 ng/dl, the sample was diluted and assessed again until the concentration was <50 ng/dl.

### 2.4. Methylation-Specific PCR (MSP)

The methylation status of the gene promoter regions was determined by MSP, and 1 *μ*g cfDNA was taken for methylation analysis. The EpiTect Bisulfite Kit (Qiagen, Germany) was used for bisulfite modification according to the manufacturer's agreement. The bisulfite-modified cfDNA was then used for MSP. The designed methylated specific sequence (M) and unmethylated specific sequence (U) primers were synthesized by Guangzhou Biotechnology Company, as listed in Table 1. PCR amplification was performed in the following conditions: 95°C for 12 min, followed by 40 cycles of 95°C for 30 seconds, 60°C for 30 seconds, and 72°C for 30 seconds. The PCR products were electrophoresed on a 1.5% agarose gel stained with ethidium bromide and observed and photographed under a gel imager.

### 2.5. Model Construction and Validation

Here, combined with sample clinical information (age, gender, and smoking history), tumor marker expression levels, and methylation frequencies of 6 genes in blood, SVM classifier was built by the python package “sklearn” to perform ten-fold cross-validation. Then, receiver operation characteristic (ROC) curves were drawn to calculate area under the curve (AUC) value to verify reliability and to evaluate the performance of the constructed diagnostic models.

The prediction performance of the model was evaluated via sensitivity (*S*_*n*_), specificity (*S*_*p*_), and accuracy (ACC) [14].

(1) $$\begin{array}{c} S_{n}=\frac{\text{TP}}{\text{TP}+\text{FN}},\\ S_{p}=\frac{\text{TN}}{\text{TN}+\text{FP}},\\ \text{ACC}=\frac{\text{TP}+\text{TN}}{\text{TP}+\text{TN}+\text{FP}+\text{FN}}. \end{array}$$

TP, TN, FP, and FN were the numbers of true positive, true negative, false positive, and false negative samples, respectively.

### 2.6. Statistical Analysis

Chi-square test was undertaken to evaluate the relationship between lung cancer patients and healthy subjects in aspects of clinicopathological features and gene methylation frequency. Owing to the serum tumor marker levels of patients and healthy subjects did not conform to the normal distribution, the data used were represented by [*M* (*P*_25_, *P*_75_)] (M: median, *P*_25_/*P*_75_: quartile), and the nonparametric Wilcoxon rank-sum test was implemented for comparison between groups. *P* < 0.05 was considered statistically significant.

### 2.7. Code Availability

The model program used to determine whether a patient has lung cancer was written by our team members and provided in the mode of open-source code (https://github.com/732618078/Classifier/blob/main/svm.py).

## 3. Results

### 3.1. Basic Information of Included Samples

The basic information and clinical features of all samples included in this study were detailed in Table 2. A total of 140 blood samples were collected, including 70 samples from lung cancer patients and 70 samples from healthy subjects. The results displayed that the distribution of age, gender, and smoking history between lung cancer patients and healthy subjects was not statistically different.

### 3.2. Detection of Tumor Markers

A total of 140 blood samples from lung cancer patients and healthy subjects were collected for analysis. The results denoted that levels of four serum tumor markers (CEA, CYFRA21-1, SCCA, and CA125) of lung cancer patients were noticeably higher than those of healthy subjects, and the difference was statistically significant, as shown in Table 3.

### 3.3. Methylation Frequencies of 6 Genes in Blood

This study identified FHIT, MGMT, P16, RASSF1A, APC, and DAPK as methylation markers of lung cancer through literature review and previous studies [9–11]. The methylation frequencies of the above 6 genes in 140 blood samples from lung cancer patients and healthy subjects were evaluated via MSP, as presented in Table 4. The results manifested that the methylation frequencies of these 6 genes in lung cancer patients were prominently higher than those in healthy subjects, and the difference was statistically significant.

### 3.4. Establishment and Validation of Diagnostic Models

For better-diagnosing lung cancer patients by clinicians, clinical information (age, gender, and smoking history), tumor marker expression levels, or methylation of risk genes was analyzed individually or collectively by a SVM classifier with 10-fold cross-validation. Afterward, several diagnostic models were constructed and validated by ROC curves (Figure 1). The results demonstrated that the combined model based on clinical information, tumor marker expression levels, and risk gene methylation levels had the best performance than the other model with only one feature, with an AUC value of 0.963, which was greater than the AUC values of the other three models (0.905, 0.805, 0.542), and *S*_*n*_, *S*_*p*_, ACC of 0.900, 0.971, and 0.936, respectively, suggesting that the combined diagnostic model of lung cancer based on all the above characteristics had a favorable performance.

## 4. Discussion

Lung cancer is the deadliest cancer that is hard to be detected in the early stage, and thus, most patients are already diagnosed in the advanced stage [15]. The current diagnostic evaluation for suspected cases of lung cancer includes tissue diagnosis, complete staging, metastasis evaluation, and patient function evaluation, whereas the false positive rate is relatively high [16]. Besides, low-dose CT screening for lung cancer can improve the early diagnosis rate, but its main weaknesses are high cost and repeated scanning that will cause certain harm to the human body [4]. Such approaches, however, have failed to diagnose lung cancer in efficacy. Therefore, probing methods that can be used to improve the diagnosis rate of lung cancer are provided with broad research prospects.

Tumor markers are important in screening, diagnosis, and efficacy evaluation of lung cancer, but their independent use is unable to identify and diagnose tumors accurately with low specificity and sensitivity [5]. Accordingly, this study attempted to establish a diagnostic model based on tumor marker levels and other characteristics of lung cancer patients. DNA methylation is a newly discovered biomarker for diagnosis, prognosis, and predictive treatment and is also one of the best-characterized, earliest, and most important [17]. Relative studies showed that the occurrence and progression of lung cancer are modulated by abnormal DNA methylation, noncoding RNAs, and histone acetylation, wherein abnormal DNA methylation is dominant. CpG island hypermethylation in the DNA promoter region of tumor suppressor genes plays a pivotal role in the occurrence and progression of lung cancer [18]. For instance, Yang et al. [19] studied the methylation frequency of DAPK promoter in NSCLC tissue and precancerous normal tissue, with the former notably higher than the latter. Yan et al. [20] found that FHIT promoter region hypermethylation is remarkably higher in NSCLC tissue than in normal lung tissue and higher in nonsmokers than smokers. FHIT hypermethylation is also associated with increased risk and worsening survival of NSCLC. Pankova et al. [21] believed that RASSF1A promoter region hypermethylation will increase the characteristics of lung cancer stem cells and elevate the risk of lung cancer metastasis progression. Moreover, tumor suppressor genes such as p16, APC, and MGMT were substantiated to be hypermethylated in lung cancer tissue [22]. These investigations indicated that the difference in methylation of tumor suppresser genes contributes to diagnosing lung cancer patients from healthy people to some degree. Hence, this study recruited 70 lung cancer patients and 70 healthy subjects for 6-gene detection via MSP, and a significant difference was found between lung cancer patients and healthy subjects in the methylation frequency of genes.

The basic idea of SVM is through mapping and constructing the classification hyperplane, to address the problem by transforming the nonlinear problem in the low-dimensional space into the linear problem in the high-dimensional space [23]. Machine learning has encountered many problems as developing, such as local minimum, nonlinearities, and dimensional disasters, as well as model selection and overfitting, while SVM can partly solve the above problems [23]. Nowadays, establish a prognostic model combining machine learning becomes an effective method for diagnosing lung cancer. For example, based on the image features collected by CT, Kavitha et al. [24] effectively segmented the lung nodules based on Fuzzy C-Means Clustering (FCM) technique and diagnosed the cancer stage based on SVM classifier. Chen et al. [25] proposed MEM-SVM by combining a modified electromagnetism-like mechanism (EM) algorithm with SVM as the classifier, and the results proved that MEM-SVM, with good diagnosis ability, can be applied as an alternative diagnostic tool for other medical tests for the early detection of brain metastasis from lung cancer. In this study, ten-fold cross-validation was carried out on the independent application of clinical characteristics (age, gender, and smoking history), tumor marker levels, and 6-gene methylation frequency, or combined application of the above three characteristics by using the SVM classifier. The verification results illustrated that the combined model was optimal with the AUC value of ROC curve at 0.963, and the *S*_*n*_, *S*_*p*_, and ACC values at 0.900, 0.971, and 0.936, respectively. These results exhibited that the combined lung cancer diagnostic model had a good performance and could well diagnose lung cancer patients from healthy people.

In conclusion, this study established a combined diagnostic model of lung cancer with favorable efficacy by SVM classifier based on sample clinical features, tumor marker levels, and 6-gene methylation frequency. This model established in this study may be of assistance to clinicians in making an accurate determination on patients with early lung cancer/pulmonary nodules, thus elevating the diagnosis rate and survival rate of lung cancer in the early stage. This study had clinical application value to some extent. While the above studies could certainly certify the accuracy of the model, there still exist inadequacies. Further work needs to be done to validate the diagnostic value of this model for lung cancer by expanding the sample volume for proof tests with multicenter combination and normalized detection.

## Figures and Tables

**Figure 1:** ROC curves of the diagnostic models.

**Table 1:** Primer sequences used in MSP.

Gene	Primer
FITH-M	Forward: 5′-GGTTTTTACGCGCGTTAGGT-3′
	Reverse: 5′-GCTCATAAAAAGCAAAATGCTCC-3′

FITH-U	Forward: 5′-GGTTTTTATGTGTGTTAGGT-3′
	Reverse: 5′-ACTCATAAAAAACAAAATACTCC-3′

P16-M	Forward: 5′-TTATTAGAGGGTGGGGCGGATCGC-3′
	Reverse: 5′-GACCCCGAACCGCGACCGTAA-3′

P16-U	Forward: 5′-TTATTAGAGGGTGGGGTGCATTGT-3′
	Reverse: 5′-CAACCCCAAACCACAACCATAA-3′

MGMT-M	Forward: 5′-TTTCGACGTTCGTAGGTTTTCGC-3′
	Reverse: 5′-GCACTCTTCCGAAAACGAAACG-3′

MGMT-U	Forward: 5′-TTTGTGTTTTGATGTTTGTAGGTTTTTGT-3′
	Reverse: 5′-AACTCCACACTCTTCCAAAAACAAAACA-3′

RASSF1A-M	Forward: 5′-GGGTTTTGCGAGAGCGCG-3′
	Reverse: 5′-GCTAACAAACGCGAACCG-3′

RASSF1A-U	Forward: 5′-GGTTTTGTGAGAGTGTGTTTAG-3′
	Reverse: 5′-CACTAACAAACACAAACCAAAC-3′

APC-M	Forward: 5′-TATTGCGGAGTGCGGGTC-3′
	Reverse: 5′-TCGACGAACTCCCGACGA-3′

APC-U	Forward: 5′-GTGTTTTATTGTGGAGTGTGGGTT-3′
	Reverse: 5′-CCAATCAACAAACTCCCAACAA-3′

DAPK-M	Forward: 5′-GGATAGTCGGATCGAGTTAACGTC-3′
	Reverse: 5′-CCCTCCCAAACGCCGA-3′

DAPK-U	Forward: 5′-GGAGGATAGTTGGATTGAGTTAATGTT-3′
	Reverse: 5′-CAAATCCCTCCCAAACACCAA-3′

**Table 2:** Basic information of included samples.

Samples	Lung cancer patients (*n* = 70)	Healthy subjects (*n* = 70)	*P*
Age			
≤60	34	42	0.17
>60	36	28	
Gender			
Male	45	36	0.12
Female	25	34	
Smoking history			
Smokers	32	22	0.21
Nonsmokers	22	26	
Former smokers	16	22	
Pathological type			
Adenocarcinoma	31	—	
Squamous cell carcinoma	39	—	
Primary lesion			
Left lung	34	—	
Right lung	36	—	
Stage			
I+II	31	—	
III+IV	16	—	
Unknown	23	—	

**Table 3:** Serum tumor marker levels of samples [*M* (*P*_25_, *P*_75_)].

Serum tumor markers	Lung cancer patients (*n* = 70)	Healthy subjects (*n* = 70)	*P*
CEA (ng/mL)	5.63 (2.83, 25.36)	1.93 (1.18, 3.51)	<0.05
CYFRA21-1 (ng/mL)	3.97 (2.50, 7.43)	1.99 (1.39, 2.49)	<0.05
SCCA (ng/mL)	1.35 (0.86, 2.70)	0.91 (0.62, 1.19)	<0.05
CA125 (U/mL)	38.21 (15.71, 85.50)	11.23 (8.00, 16.12)	<0.05

**Table 4:** Methylation frequencies of 6 genes in included samples.

Methylation frequency	Lung cancer patients (*n* = 70)	Healthy subjects (*n* = 70)	*P*
*FHIT*			
Methylation	33	1	<0.05
Nonmethylation	37	69	
*P16*			
Methylation	14	4	<0.05
Nonmethylation	56	66	
*MGMT*			
Methylation	7	1	<0.05
Nonmethylation	63	69	
*RASSF1A*			
Methylation	26	5	<0.05
Nonmethylation	44	65	
*APC*			
Methylation	33	7	<0.05
Nonmethylation	37	63	
*DAPK*			
Methylation	24	3	<0.05
Nonmethylation	46	67	

## Data Availability

The data used to support the findings of this study are included within the article. Any additional data and materials if required could be made available from the corresponding author on reasonable request.
